# Efficacy and Safety of Immunosuppressant Therapy for Noninfectious Uveitis: A Systematic Review and Meta-Analysis

**DOI:** 10.1155/2021/1933604

**Published:** 2021-09-04

**Authors:** Haihong Zuo, Wei Zhang, Yuqing Yan

**Affiliations:** ^1^Department of Ophthalmology, Tianjin Haihe Hospital, Tianjin 300350, China; ^2^Department of Stomatology, Tianjin Haihe Hospital, Tianjin 300350, China

## Abstract

**Objective:**

To analyze efficacy and safety of immunosuppressant therapy for noninfectious uveitis.

**Methods:**

A network search of PubMed, ResearchGate, and EMBASE databases was conducted for relative literature and studies from the inception of each database to April 2021. Primary outcomes were efficacy and time to treatment failure of immunosuppressant for noninfectious uveitis. Secondary outcome was incidence of adverse events (AEs). Cochrane risk of bias tool was used to assess risk of bias of included studies. Fixed effects model or random effects model was implemented to assess statistical heterogeneity. Subgroup analysis was employed to analyze heterogeneous sources.

**Results:**

Eight studies were deemed eligible for inclusion with a total of 848 patients. Six studies were randomized controlled trials (RCTs). Among them, a single-blind RCT had relatively high measurement bias and performance bias. Immunosuppressant presented favorable efficacy for noninfectious uveitis than placebo, and RR was 1.43 (95% CI: 1.12-1.82). Immunosuppressant for noninfectious uveitis prolonged the time before failure, and HR was 0.43 (95% CI: 0.32-0.54). AEs increased after immunosuppressant was applied. Compared with immunosuppressant, RR of AEs with placebo was 0.88 (95% CI: 0.71-1.08).

**Conclusion:**

Immunosuppressant contributed to controlling progression of noninfectious uveitis to some extent. Compared with placebo, it increased incidence of AEs. More studies with low heterogeneity are warranted for stronger evidence in clinical.

## 1. Introduction

Noninfectious uveitis may be induced by various diseases, containing systemic or idiopathic inflammatory diseases [1]. Persistent infiltration in conditions with inflammatory cells is responsible for retinal damage and blindness [2]. In the past, the main first-line treatment for noninfectious uveitis was administration of topical or systemic corticosteroids. Recently, a therapeutic approach with immunosuppressant drugs has gradually been adopted by clinicians. The treatment for noninfectious uveitis is a long-term process, and thus, the conventional approach is obviously not suitable for patients who are intolerant to long-term application of corticosteroids [3]. Immunosuppressant, especially tumor necrosis factor- (TNF-) *α* monoclonal antibody, is applied in refractory noninfectious uveitis with encouraging outcomes in some, but not all, cases [4]. Hence, a systematic review on clinical efficacy and safety of immunosuppressants in treatment for noninfectious uveitis is warranted.

At present, some immunosuppressants are used in clinical practice, including methotrexate (an antimetabolite), mycophenolate mofeti, adalimumab, and interferon-*α*2a [5]. A study [6] from South Korea displayed that adalimumab has a favorable clinical efficacy for refractory uveitis. Another study unraveled the use of infliximab after adalimumab failure in pediatric noninfectious uveitis [7]. Besides, after being treated with adalimumab, best-corrected visual acuity (BCVA) of patients is improved [8]. A study on drug retention rate (DRR) and drug retention time (DRT) of adalimumab in uveitis manifested that discontinuation in 151 patients is composed of loss of efficacy in 74 patients and adverse events (AEs) in 34 patients [9].

This systematic review and meta-analysis attempted to evaluate clinical efficacy and safety of immunosuppressant therapy for noninfectious uveitis and to provide references for further clinical therapy.

## 2. Methods

### 2.1. Study Selection

In this study, study selection strategy was designed following Preferred Reporting Items for Systematic Reviews and Meta-Analysis (PRISMA) [10]. A network search of PubMed, ResearchGate, and EMBASE databases was conducted for relative literature and studies from inception of each database to April 2021. Search keywords included “noninfectious uveitis,” “refractory uveitis,” “autoimmune uveitis,” “idiopathic uveitis,” “immunomodulator,” “immunity inhibitor,” “tumor necrosis factor-alpha inhibitors,” “adalimumab,” and “infliximab.” Both full names and abbreviations of proper nouns were searched. Two investigators independently performed study selection. Titles, abstracts, and full texts were screened. Titles and abstracts were scanned to exclude apparently ineligible studies, and full text of potentially eligible studies was assessed for final inclusion by the two investigators independently. While screening, any discrepancies were resolved by discussion by two investigators or final judge by a third investigator. Cochrane risk of bias tool [11] was used to assess risk of bias of included randomized controlled trials (RCTs).

Included criteria are as follows: (1) research object: noninfectious uveitis; (2) one patient cohort with noninfectious uveitis was treated with immunosuppressant drugs; (3) the study reported at least one of the following items: efficacy, treatment failure time, and incidence of AEs, for evaluation of clinical efficacy indicators of immunosuppressive drugs in the treatment of noninfectious uveitis (efficacy indicator forms can be rate ratio (RR) or hazard ratio (HR)); and (4) evaluation on safety of drugs.

Exclusion criteria are as follows: (1) non-English literature; (2) nonfull text; (3) outcomes related to efficacy and safety cannot be converted into RR or HR; (4) primary outcome was dose-limiting toxicity of drugs; (5) sample cohorts were two different types of noninfectious uveitis (e.g., acute noninfectious uveitis vs. chronic noninfectious uveitis).

### 2.2. Data Extraction

The following information was extracted: (1) first author; (2) year of publication; (3) type of study; (4) interventional method; (5) sample size; (6) primary outcomes: (a) efficacy (determination was made according to change of the best corrected visual acuity (logarithm of minimum resolution angle) of each eye, time of optical coherence tomography (OCT), change of anterior chamber cell level of each eye, change of vitreous fog level of each eye, percentage of change of the central retinal thickness of each eye, change of comprehensive score of NEI Visual Function Questionnaire (VFQ-25), and other indicators) and (b) time to treatment failure; and (7) second outcome: incidence of AEs. Time to treatment failure was expressed as HR (95% CI). Data extraction was also conducted independently by the two investigators.

### 2.3. Statistical Analysis

Cochrane risk of bias assessment was performed on RevMan (version 5.4). In Stata/MP (version 16.0), statistical analyses of relative indexes were carried out. Cochran's *Q* test and *I*^2^ statistic were implemented to detect statistical heterogeneity of efficacy, time to treatment failure, and AEs between studies. Efficacy and incidence of AEs were included in the analysis as measurement data. A fixed effects model was used on the assumption that there was no statistical heterogeneity between studies. *I*^2^ statistic > 50% or *p* < 0.1 was considered statistical heterogeneity; random effects model was utilized for retesting. Time to treatment failure was assessed for the statistical difference by random effects model. Subgroup analysis was carried out on indexes with *I*^2^ statistic > 50% or *p* < 0.1 to analyze heterogeneous sources.

## 3. Results

### 3.1. Literature Retrieval

Following the study selection strategy, 3116 articles were initially retrieved, and 436 duplicate articles were excluded. After two investigators scanned titles and abstracts of articles independently, 2623 apparently ineligible studies were excluded. Among 57 potentially eligible studies, 23 articles that were not available for full text were excluded. Then, the two investigators conducted content reviews on 34 articles independently, and finally, 7 studies were deemed eligible for inclusion (Figure 1).

### 3.2. Baseline Characteristics of Included Literature and Results of Cochrane Risk of Bias Assessment

A total of 8 articles [12–19] were deemed eligible for inclusion in this study. A total of 848 patients (intervention group: *n* = 465) were enrolled for analysis. Five investigations were double-blind RCTs: one is prospective study and one is a retrospective study (Table 1). The results of Cochrane's risk of bias displayed that among 6 RCTs, a single-blind RCT had a relative high measurement bias and performance bias (Figures 2(a) and 2(b)).

### 3.3. Heterogeneity Analysis of Primary Outcomes and Secondary Outcome

#### 3.3.1. Statistical Heterogeneity Analysis of Primary Outcomes

The included 8 studies all reported clinical efficacy of immunosuppressant drugs for noninfectious uveitis, whereas there was moderate statistical heterogeneity among them (Figure 3(a)). Forest plot of statistical heterogeneity analysis on efficacy showed *I*^2^ = 64.3%, *p* = 0.01. RR of immunosuppressant therapy for noninfectious uveitis was 1.43 (95% CI: 1.12-1.82), suggestive of better efficacy in the immunosuppressant group than in the placebo group.

Three studies reported the time to treatment failure. Random effects model displayed that there was moderate statistical heterogeneity among them (Figure 3(b)) (*I*^2^ = 65.4%, *p* = 0.056). HR of time to treatment failure was 0.43 (95% CI: 0.32-0.54), indicating that the time before failure was prolonged with immunosuppressant therapy.

#### 3.3.2. Statistical Heterogeneity Analysis of Secondary Outcome

Among 8 included studies, 3 reports about AEs could be subjected to quantitative analysis. Forest plot of statistical heterogeneity analysis on AEs disclosed that there was no statistical heterogeneity among them (Figure 4) (*I*^2^ = 0.0%, *p* = 0.541). RR of AEs with placebo was 0.88 (95% CI: 0.71-1.08). Hence, immunosuppressant increased AEs.

### 3.4. Subgroup Analysis

According to Section 3.3.1, this study analyzed heterogeneous sources of efficacy. Based on therapeutic regimens, 7 trials were divided into two subgroups (adalimumab vs. placebo and nonadalimumab vs. placebo). The results of heterogeneous subgroup analysis unveiled that the nonadalimumab vs. placebo group may be potentially heterogeneous sources (Figure 5).

## 4. Discussion

Two RCTs (trials SYCAMORE and ADJUVITE) confirmed clinical efficacy of anti-TNF-*α* antibody for uveitis associated with juvenile idiopathic arthritis (JIA) [15, 20], and they were also included in this study. Meta-analysis illustrated that compared with placebo or other drugs, immunosuppressant therapy for noninfectious uveitis had clinical efficacy to some extent, whereas there was moderate heterogeneity among studies. Due to the lack of evidence-based evidence with high quality, clinical effect of adalimumab for noninfectious uveitis cannot be defined accurately. Besides, relative studies believed that some patients who suffer uveitis associated with juvenile idiopathic arthritis (JIA) generate permanent anti-adalimumab antibodies after adalimumab treatment, which affects clinical efficacy of adalimumab for those patients, while administration with other immunosuppressants contributes to reducing generation of anti-adalimumab antibodies [21]. Although some patients achieved treatment failure with immunodepressants [22], our results disclosed that compared with placebo, monotherapy or combined therapy of immunosuppressant could prolong the time to treatment failure in effect. Nonetheless, there was a certain degree of statistical heterogeneity among the included studies, and unfortunately, we failed to investigate potentially statistical heterogeneity sources from the extracted information in the research.

*Guidance on Noncorticosteroid Systemic Immunomodulatory Therapy in Noninfectious Uveitis* proposed that it is possible to use noncorticosteroid systemic immunomodulatory drugs to control persistent or noninfectious uveitis with severe inflammation, thereby preventing complications that cause structural damage to the eyes [23]. Meta-analysis of safety of immunosuppressant therapy for noninfectious uveitis revealed that compared with placebo, immunosuppressant increased incidence of AEs. Long-term dependence on immunosuppressants may increase the risk of infection, though their association has not been proved yet in the POSUT project [24]. Since the included studies performed incidence of AEs in different formats, this study only carried out a meta-analysis on three studies. Besides, this study did not report in detail whether the incidence of different types of AEs (injection site reaction, infection, etc.) is associated with immunosuppressant drugs. In the guideline, it was also suggested that immunosuppressant drug and corticosteroid reduction can be applied in subsequent treatments if the patient does not respond to standard treatments [23]. A more comprehensive and detailed systematic review and meta-analysis are required to assess safety of immunosuppressant drugs for noninfectious uveitis.

In conclusion, this study systematically reviewed efficacy and safety of immunosuppressant drugs for noninfectious uveitis. Immunosuppressants contributed to controlling noninfectious uveitis, but their safety needs more evidence-based supports.

## Figures and Tables

**Figure 1:** Flow chart of study selection.

**Figure 2:** Evaluation on quality of RCTs with Cochrane risk of bias tool.

**Figure 3:** Heterogeneity analysis of primary outcomes. (a) Forest plot of heterogeneity analysis on efficacy. (b) Forest plot of heterogeneity analysis on time to treatment failure.

**Figure 4:** Heterogeneity analysis of the incidence of AEs.

**Figure 5:** Forest plot of subgroup heterogeneity analysis of efficacy according to therapeutic regimens.

**Table 1:** Baseline information of included literature.

Author	Year	Type of study	Intervention (treatment vs. control)	Patients (treatment/control)	Female (treatment/control)	Efficacy (yes/no) treatment vs. control
Nguyen et al.	2016	RCT, DB	Adalimumab vs. placebo	115/111	66/72	70/45 vs. 50/61
Jaffe et al.	2016	RCT, DB	Adalimumab vs. placebo	—	—	—
Ramanan et al.	2017	RCT, DB	Adalimumab vs. placebo	60/30	47/23	44/16 vs. 12/18
Quartier et al.	2017	RCT, DB	Adalimumab vs. placebo	16/15	15/13	9/7 vs. 3/12
Cecchin et al.	2018	Prospective study	Adalimumab vs. infliximab	95/59	16/15	57/38 vs. 12/47
Heissigerová et al.	2018	RCT, DB	Sarilumab vs. placebo	38/20	23/13	29/9 vs. 15/5
Rathinam et al.	2019	RCT, SB	Methotrexate vs. mycophenolate mofetil	107/109	75/60	64/43 vs. 56/53

RCT: randomized controlled trial; DB: double-blind; SB: single-blind; DMARDs: disease-modifying antirheumatic drugs.

## Data Availability

No data were used to support this study.
